# An Untargeted Lipidomics Study of Acute Ischemic Stroke with Hyperglycemia Based on Ultrahigh-Performance Liquid Chromatography-Mass Spectrometry

**DOI:** 10.1155/2022/8332278

**Published:** 2022-08-26

**Authors:** Jia Guo, Hailan Wang, Xin Jiang, Yan Wang, Zhihao Zhang, Qingbin Liao, Jia Xu

**Affiliations:** Department of Geriatrics, Dadukou District People's Hospital, Chongqing 400084, China

## Abstract

Patients with type 2 diabetes have twice as much of the risk of acute ischemic stroke (AIS) occurrence as healthy individuals, and the AIS patients with type 2 diabetes have a higher risk of death and a poorer prognosis. This study was to investigate the interrelationship between hyperglycemia and AIS and provided a reference for blood glucose management of AIS patients. The blood glucose level of AIS patients of the present study was controlled by insulin below 180 mg/dL (standard group) and between 80 and 130 mg/dL (management group). And the fasting venous blood samples were collected for determination of blood glucose level, homeostasis model assessment of insulin resistance (HOMA-IR), peptide C, and basal insulin level. Furthermore, lipids of the blood samples were detected using metabolomics, so as to clarify the similarities and differences in metabolic patterns in AIS patients with diabetes after the intervention of different glycemic strategies. The results revealed that compared to the standard group, the blood glucose level and HOMA-IR in the management group were significantly decreased, and levels of peptide C and basal insulin level were greatly increased. Through lipidomics detection, 83, 50, and 44 types of significantly upregulated differential lipids were detected in the standard vs. normal groups, the standard vs. management groups, and the management vs. normal groups, respectively, with triacylglycerol dominated. This study preliminarily revealed metabolic differences among AIS patients with hyperglycemia after different blood glucose intervention methods, hoping to provide a theoretical basis for clinical prevention and treatment of this disease.

## 1. Introduction

Acute ischemic stroke (AIS) is recognized as a serious brain vessel disease with extremely high fatality and disability rates [1], and the risk of AIS in patients with type 2 diabetes is about twice that of healthy individuals [2]. Diabetes treatment can effectively reduce the severity of AIS and improve the prognosis of patients [3]. Glucose control is a challenge during the acute care of AIS patients currently, which contributes to neuroprotection according to several studies [4]. Despite the fact that hyperglycemia is regarded as a risk factor for AIS patients, doubts on the effectiveness of blood sugar control has been raised by some scholars [5]. Research on Chinese AIS patients has indicated that blood sugar control below 200 mg/dL is necessary [6]. Some researchers have proposed that neuroprotective measures for AIS patients with hypoglycemia should be based on vascular thrombolysis and imaging-assisted classification [7]. Most previous studies on blood glucose in AIS patients have focused on the detection of blood glucose, high- and low-density lipoproteins, and the causal relationship between AIS and hyperglycemia is still unclear. In recent years, significant progress has been made in the metabolomics of small molecules. Typically, an untargeted metabolomics approach is aimed at characterizing global metabolism and quantifying hundreds or thousands of small- and medium-sized molecules, mainly in urine, serum, and tissue extracts [8]. Untargeted lipidomics can fully collect information in metabolic networks, thereby depicting a more comprehensive profile of metabolic mechanisms of disease. As the continuous improvement of databases, untargeted metabolomics research based on mass spectrometry is more convenient with a wider application than the method based on nuclear magnetic resonance [9].

Unluckily, previous research and the current clinical treatment protocols are not complete; it is of great practical significance to clarify the causal relationship between AIS and hyperglycemia and to investigate blood glucose control in the acute phase of AIS patients. In light of previous research findings and treatment guidelines, the present project classified the AIS patients into three groups: AIS normal group with normal glucose, AIS diabetes-standard group, and AIS diabetes-management group. In terms of hypoglycemic measures, the management group was treated using a strict blood sugar control scheme and the standard group was treated using a standard blood sugar control scheme. Simultaneously, based on general blood biochemistry, metabolomics was applied to detect small molecular substances in patients and to explore the differences in lipid metabolism of AIS diabetic patients in each group at the molecular level.

## 2. Materials and Methods

### 2.1. Instruments, Reagents, and Materials

The instruments included the 1290 ultrahigh-performance liquid chromatography instrument (UHPLC) from Agilent, USA; Q Exactive Focus High-Resolution Mass Spectrometer, Heraeus Fresco 17 Centrifuge, and NanoDrop One Microplate Reader from Thermo Fisher, USA; and SYNCHRON LX-20 Biochemistry Analyzer from Beckman Coulter, USA. The reagents and materials included insulin kit (RX104930H) and serum peptide C kit (RX106372H). Both were purchased from Quanzhou Ruixin Biotechnology Co., Ltd. LC-MS, methanol, acetonitrile, ammonium formate, and dichloromethane were purchased from CNW, Germany.

### 2.2. Test Grouping

The patients with fasting blood glucose ≥ 6.1 mmol/L were divided into the hyperglycemia group, and those with fasting blood glucose < 6.1 mmol/L were divided into the normal group. The hyperglycemia group was subdivided into standard and management groups according to their history of diabetes. There were a total of 54 patients included, with 18 cases in each of the described three groups: AIS normal group with normal glucose, AIS diabetes-standard group, and AIS diabetes-management group, respectively. The inclusion criteria are shown in Table 1. Blood glucose of the patients was measured and recorded every 8 hours. Patients in the AIS normal group with normal glucose were given no treatment; patients in the standard group were injected with insulin once the blood sugar level increased above 180 mg/dL, and the dose was increased if the target concentration was not reached within 12 h; the blood sugar concentration of the management group was strictly controlled within the 80-130 mg/dL range using insulin.

### 2.3. Determination of Blood Biochemical Indicators

The patients were treated with different management measures for blood sugar control, and fasting venous blood was collected 24 h later for the detection of blood biochemical indicators. Fasting blood glucose levels were detected using the SYNCHRON Biochemical Analyzer. The basal level of insulin and the concentration of C-peptide were detected using the test kit, performed strictly in accordance with the instructions of use. Insulin resistance index (HOMA‐IR) = (fasting glucose level × basal insulin level)/22.5.

### 2.4. Sample Pretreatment

The complete blood samples were performed centrifugation at 4000*g* 4°C for 15 min, and 30 *μ*L of the supernatant was aspirated to a new tube for further extraction. Following the addition of 90 *μ*L of precooled methanol-acetonitrile (*v*/*v* = 1 : 1) to the serum, the solution was vortexed for 1 min and kept in an ice-water bath for 15 min. The mixed solution was centrifuged at 12,000*g*, 4°C for 15 min, and 100 *μ*L of the supernatant was collected and kept in a sample vial for subsequent analysis.

### 2.5. LC-MS Sample Loading Detection

The samples were analyzed by ultrahigh-performance liquid chromatography-mass spectrometry (UHPLC-MS) technique, and the vacuum-dried solids were redissolved using 100 *μ*L of 50% methanol. After centrifugation at 12,000*g* 4°C, the supernatant was transferred to a sample vial. Chromatographic separation was performed using an ultrahigh-performance liquid chromatography system packed with a BEHC18 column (2.1 mm × 100 mm, 1.7 *μ*m). The prepared sample volume was 5 *μ*L, mobile phase A was 0.1% formic acid-acetonitrile, and mobile phase B was 0.1% formic acid-water. The flow rate was 0.35 mL/min, and the column temperature was 40°C. The analysis was conducted with chromatographic gradient as follows: 0-0.5 min, 1% A; 0.5-3.5 min, 1-53% A; 3.5-7.5 min, 53-70% A; 7.5-9 min, 70-90% A; 9-13 min, 90% A; 13.1-15 min, and back to 1% A. To ensure a steady system, the quality control samples were used at the beginning and end of each analysis. Mass spectrometry data were collected using ESI source in positive and negative ion modes, and the specific scanning parameters were capillary voltage 4 kV in positive ion mode, 3.5 kV in negative ion mode, atomizing gas temperature at 330°C, atomizing gas flow rate 10 L/min, splitting voltage at 100 V, screening voltage at 65 V, scanning range *m*/*z* 70-1100, and scanning speed 1.5 scan/sec.

### 2.6. Bioinformatics Analysis

The LC-MS data preprocessing included peak detection, extraction, alignment, and integration which were mainly implemented using the xcms toolkit of R platform. The bandwidth was set to 15 sec, the peak broadening 5-30 sec, and other parameters default. The preprocessed data were imported into EZinfo software in matrix for principal component analysis (PCA) and orthogonal partial least squares-discriminant analysis (OPLS-DA); and the data were imported into MetaboAnalyst for hierarchical clustering analysis (HCA). Kruskal-Wallis tests, Student's *t*-tests, and logistic regression analysis were all implemented using the R software to assess the influence of confounding factors.

### 2.7. Statistical Analysis

The blood biochemical index data were statistically analyzed using GraphPad Prism 9.0 software, and the results were expressed as mean ± standard deviation (SD). One-way ANOVA was applied for significant analysis; when *p* < 0.05, the difference was considered significant.

## 3. Results

### 3.1. Differences in Blood Biochemical Indexes among Groups

The fasting glucose levels and HOMA-IR levels of the standard group were significantly higher than those of the normal group (*p* < 0.01) and the management group (*p* < 0.05) (Figures 1(a) and 1(b)), while the serum peptide C and basal insulin levels were markedly lower than those of the control and management groups (*p* < 0.01) (Figures 1(c) and 1(d)).

### 3.2. Multivariate Statistical Analysis

Sample PCA was conducted using multivariate statistics.  Figure 2(a) presents *R*^2^*X* = 0.647 > 0.4, and QC was clustered together, indicating that the instrument was stable during the sample collection and the data reproducibility was satisfactory which were applicable for subsequent analysis. PCA revealed that normal vs. standard, normal vs. management, and management vs. standard groups had the tendency to separate and were clearly clustered into two groups to be distinguished effectively, indicating that there was a significant difference (Figures 2(b)–2(d)). The scatter point diagram of the OPLS-DA model indicated evident separation of the normal group and the AIS diabetic group. In Figures 3(a)–3(c), *R*^2^*X* were 0.575, 0.534, and 0.546; *R*^2^*Y* were 0.991, 1.000, and 0.998; *Q*^2^ were 0.904, 0.981, and 0.913, indicating that the predicted probabilities of the model were 90.4%, 98.1%, and 91.3%, respectively. Permutation test was performed on the model also with the results presented in Figures 4(a)–4(c). The *y*-axis intercept of *Q*^2^ in each group was all below 0, implying that the model had been fitted and differential metabolites could be screened accordingly.

### 3.3. Identification of Differential Lipid Metabolism

Through the above analysis, combined with the statistical results of univariate and multivariate analysis, differential metabolites were screened out. To present a better visualization of the differences among groups, a volcano plot (Figures 5(a)–5(c)), cluster analysis (Figures 6(a)–6(c)), and a lipid group bubble plot (Figures 7(a)–7(c)) were constructed based on the identified lipid metabolites, and there were substantial differences in lipid products and evident hierarchical clustering among each of the groups. A total of 83 differentially upregulated lipid metabolites were screened from the standard group compared with the normal group based on variable importance in projection (VIP) > 1, *p* < 0.05 of *t*-tests, and fold change (FC) > 2 of the maximum difference fold. Eighty-three significantly upregulated differential lipid metabolites were screened from the standard group compared with the normal group and were classified into nine categories. They were divided into nine categories: acylcarnitine (Acar), diacylglycerol (DAG), diacylglyceryl trimethylhomoserine (DGTS), hexosylceramide nonhydroxy fatty acid-sphingosine (HexCer/NS), lysophosphatidylcholine (LPC), lysophosphatidylethanolamine (LPE), phosphatidylcholine (PC), sulfur hexosylceramide hydroxy fatty acid (SHexCer), and triacylglycerol (TAG). A total of 50 differentially upregulated lipid metabolites were screened from the standard group compared with the management group, which were classified into eight categories: cholesteryl ester (CE), ceramide nonhydroxy fatty acid-dihydrosphingosine (Cer/NDS), ceramide nonhydroxyl fatty acid-sphingosine (Cer/NS), HerCer/NS, LPC, PC, sphingomyelin (SM), and TAG. A total of 44 differentially upregulated lipid metabolites were sorted out from the management group compared with the normal group, which were grouped into eight categories: acyl glucuronic acid glycolipid (AcylGlcADG), CE, DGTS, HerCer/NS, LPC, PC, SHexCer, and TAG. TAG dominated the differential metabolites screened from the three groups, and the specific differential metabolites are shown in Table 2.

## 4. Discussion

AIS has a very high morbidity and mortality, and it is often accompanied by hyperglycemia in the acute phase [10]. Many studies have indicated the interrelationship between hyperglycemia and poor clinical outcomes in AIS patients [11]. At present, there is no unified standard for the definition of hyperglycemia after AIS onset at home and abroad, and the majority of scholars set the blood glucose threshold as 6-8 mmol/L [12, 13]. Increasing evidence has revealed that hyperglycemia increases infarct size, risk of hemorrhagic transformation after reperfusion, and mortality in AIS patients, and there is a linear relationship between post-AIS hyperglycemia and poor clinical outcomes [14]. Some researchers have pointed out that there is a high mortality rate within 72 hours of onset for AIS patients with the admission blood glucose greater than 7.9 mmol/L [15]. Hyperglycemia adversely affects the prognosis of AIS patients, and the majority of cases develop cerebral infarction with large vessel occlusion.

Fasting glucose levels are commonly used clinical indicators for monitoring the degree of glucose metabolism and blood glucose control, which is an essential part for the prevention and treatment of diabetes complications [16]. Peptide C levels indicate if the secretory function of *β* cells is working well or not in the body, and it can be used as a guiding indicator for the differentiation of diabetic patients and the identification of hypoglycemia [17]. Some present studies have shown that C-peptide has a good protective effect on diabetes and its complications. It protects the functions of *β* cells and stimulates the direct secretion of insulin, thereby reducing high glucose load and relevant hyperglycemic effect on *β* cells and other cells of the entire body. Peptide C can also inhibit reactive oxygen species produced by excess glucose and fat and protect the functions of *β* cells through antioxidant pathways [18]. Insulin is an indispensable factor in the control of blood glucose levels, which regulates the expression and transport of glucose transporters in different types of tissues. Hence, insulin insensitivity results in increased intestinal glucose absorption, increased renal glucose reabsorption, and impaired peripheral tissue glucose uptake causing hyperglycemia. Conversely, high blood glucose level further reduces insulin sensitivity, creating a vicious circle [19]. Insulin resistance and *β* cell function failure are the two main causes of type 2 diabetes. As the disease progresses, more serious basal insulin secretion disorder occurs, so correcting insulin resistance is the key to controlling blood glucose levels [20].

The blood biochemical test findings indicated that the levels of fasting blood glucose and HOMA-IR in the standard group were markedly higher than those in the normal group and the management group, whereas the serum peptide C concentration and basal insulin level were substantially lower than those in the normal group and the management group. The results revealed that decreased basal insulin level impaired the absorption and processing ability of glucose. Fat cells and muscle cells cannot effectively utilize glucose substances, and liver cells fail to regulate glycogen decomposition and gluconeogenesis, resulting in an evident increase in blood glucose concentration [21, 22]. Conversely, after strict blood glucose management, the indicators in the management group differed largely from those in the standard group, suggesting that the treatment option was effective. The UHPLC-MS detection results revealed that triacylglycerol, the differential lipid metabolites in the standard group compared with the normal group, the management group compared with the normal group, and the standard group compared with the normal group were all markedly upregulated. Normally, insulin inhibits the lipolysis of triacylglycerol in adipose tissue. In the presence of insulin resistance, increased lipolysis produces more free fatty acids, thereby inhibiting the antilipolytic effect of insulin. As more free fatty acids enter the liver, hepatic triacylglycerol synthesis increased, resulting in hypertriglyceridemia [23], decreased cerebral hemodynamic indicators, and increased risk of stroke. It is an independent risk factor for stroke, suggesting that elevated triacylglycerol is closely related to the occurrence of stroke [24].

Taken together, the experimental findings revealed that insulin injection could reduce blood glucose levels and correct the insulin resistance levels in patients with AIS diabetes mellitus. However, as diabetic patients are not sensitive to insulin, strict blood sugar management regimens are more effective in lowering the glucose levels in AIS diabetic patients. Additionally, triacylglycerol is also an independent factor affecting the occurrence of stroke and diabetes. Lower blood triacylglycerol levels can reduce the antilipolysis effect of decomposed fatty acids on insulin and better exert hypoglycemic effect of insulin, allowing to resume normal glucose levels. Meanwhile, it can reduce the effect of triacylglycerol on hemodynamics and minimize the risk of stroke.

## 5. Conclusion

The use of strictly managed glycemic control strategy can reduce blood glucose levels, insulin resistance levels in patients with AIS diabetes mellitus. Triacylglycerol is an independent risk factor for stroke occurrence, and lowering blood triacylglycerol levels can prevent elevated blood glucose and reduce the probability of stroke. Our study provides a theoretical reference for the prevention and treatment of hyperglycemic AIS.

## Figures and Tables

**Figure 1:** Results of blood biochemical indicators: (a) fasting blood glucose level; (b) HOMA-IR; (c) peptide C level; (d) basal insulin level. ^∗^*p* < 0.05 and ^∗∗^*p* < 0.01.

**Figure 2:** Scatter point diagrams based on PCA: (a) standard, management, and normal groups and QC samples; (b) normal group vs. standard group; (c) normal group vs. management group; (d) management group vs. standard group. Red dots represent the normal group, purple dots represent the standard group, blue dots represent the management group, and yellow dots represent QC.

**Figure 3:** Scatter point diagrams based on OPLS-DA: (a) normal group vs. standard group; (b) standard group vs. management group; (c) management group vs. normal group. Red dots represent the normal group, purple dots represent the standard group, and blue dots represent the management group.

**Figure 4:** Permutation test plots based on OPLS-DA: (a) normal group vs. standard group; (b) standard group vs. management group; (c) management group vs. normal group.

**Figure 5:** Volcano maps of differential lipid screening: (a) normal group vs. standard group; (b) standard group vs. management group; (c) management group vs. normal group.

**Figure 6:** Heat maps of hierarchical cluster analysis: (a) normal group vs. standard group; (b) standard group vs. management group; (c) management group vs. normal group.

**Figure 7:** Bubble plots of lipid analysis: (a) normal group vs. standard group; (b) standard group vs. management group; (c) management group vs. normal group.

**Table 1:** Criteria for inclusion and exclusion of AIS subjects.

Inclusion criteria	Exclusion criteria
(I) AIS diagnosed by brain CT or MRI (II) The time from onset to hospital admission was within 24 hours (III) No history of stroke (IV) Clear consciousness (V) The patients and their family members agreed and signed the informed consent, which was approved by the ethics committee of this hospital	(I) Patients in a critical condition or combined with severe trauma and uncooperative with examinations (II) Patients with severe cardiopulmonary disease requiring complex and comprehensive testing and treatment (III) Patients with respiratory diseases or liver and kidney failures (IV) Patients with history of mental illness (V) Patients under hormone or immune stimulant administration in recent time or currently (VI) Patients who discontinued the study

Abbreviations: CT: contrast-enhanced cerebral computed tomography; MRI: magnetic resonance imaging.

**Table 2:** Differences of lipid metabolites between groups.

Number	Standard vs. normal	Standard vs. management	Management vs. normal
1	Acar(20:1)	CE(18:1)	AcylGlcADG(22:1/22:1/14:0)
2	DAG(16:0/18:0)	CE(18:2)	CE (18:2)
3	DGTS(19:0/26:2)	CE(18:3)	CE (18:3)
4	DGTS(2:0/17:1)	CE(20:5)	DGTS(2:0/17:1)
5	DGTS(2:0/21:2)	CE(22:4)	DGTS(2:0/21:2)
6	DGTS(27:0/18:1)	Cer/NDS(d18:0/24:0)	DGTS(27:0/18:1)
7	HexCer/NS(d18:1/16:1)	Cer/NS(d18:1/24:2)	HexCer/NS(d18:1/16:1)
8	LPC(14:0)	HexCer/NS(d20:3/36:1)	LPC(14:0)
9	LPC(15:1)	LPC(20:4)	LPC(15:1)
10	LPC(18:1)	PC(14:0e/20:4)	LPC(18:1)
11	LPC(18:3)	PC(14:0e/21:0)	LPC(18:3)
12	LPC(19:0)	PC(14:0e/23:0)	LPC(19:0)
13	LPC(19:1)	PC(14:0e/24:0)	LPC(19:1)
14	LPC(20:0)	PC(16:1e/22:6)	LPC(20:0)
15	LPC(20:1)	PC(18:0e/22:3)	LPC(20:1)
16	LPC(20:5)	PC(19:1/20:4)	LPC(20:2)
17	LPC(24:1)	PC(20:3/20:3)	LPC(20:3)
18	LPE(16:0)	SM(d14:0/24:0)	LPC(20:4)
19	LPE(18:2)	SM(d14:0/26:0)	PC(14:0e/20:4)
20	LPE(20:4)	SM(d14:0/27:0)	PC(14:0e/4:0)
21	LPE(22:5)	SM(d14:0/30:1)	PC(14:1e/4:0)
22	PC(11:0/22:2)	TAG(12:1/19:1/19:1)	PC(14:1e/6:0)
23	PC(11:0/26:2)	TAG(13:0/13:0/21:4)	PC(16:1e/22:6)
24	PC(12:0/26:1)	TAG(13:0/13:0/21:5)	PC(18:2/18:2)
25	PC(14:0/22:5)	TAG(13:0/18:2/18:2)	PC(18:3/18:3)
26	PC(14:0e/20:4)	TAG(13:0/21:2/21:2)	PC(20:4/20:4)
27	PC(14:0e/22:3)	TAG(13:1/18:4/18:4)	PC(24:4/18:5)
28	PC(14:0e/4:0)	TAG(13:1/21:1/21:1)	PC(3:0/18:4)
29	PC(14:1e/4:0)	TAG(14:0/18:2/20:5)	SHexCer(d18:1/16:0)
30	PC(14:1e/6:0)	TAG(14:1/14:1/22:3)	TAG(12:0/22:0/22:0)
31	PC(16:2/22:6)	TAG(15:1/19:0/21:2)	TAG(12:1/12:1/19:5)
32	PC(18:2/18:2)	TAG(16:0/16:2/22:6)	TAG(12:1/22:0/22:0)
33	PC(18:3/18:3)	TAG(16:0/20:4/20:4)	TAG(13:0/13:0/16:0)
34	PC(20:1/20:1)	TAG(16:1/16:1/22:5)	TAG(13:1/21:1/21:1)
35	PC(21:2/21:2)	TAG(16:1/18:3/20:4)	TAG(16:0/18:1/22:0)
36	PC(22:6/22:6)	TAG(16:2/18:2/18:2)	TAG(16:0/20:0/20:0)
37	PC(24:4/18:5)	TAG(17:0/18:5/22:0)	TAG(16:0/22:1/22:1)
38	SHexCer(d18:1/16:0)	TAG(17:1/19:1/19:1)	TAG(18:0/18:0/20:0)
39	TAG(12:0/12:0/22:7)	TAG(18:0/20:4/22:6)	TAG(18:0/18:0/20:1)
40	TAG(12:0/14:0/20:2)	TAG(18:1/18:2/20:4)	TAG(18:0/18:0/22:0)
41	TAG(12:0/16:0/18:1)	TAG(18:1/18:2/22:4)	TAG(18:0/18:0/22:1)
42	TAG(12:0/22:0/22:0)	TAG(18:1/20:4/22:5)	TAG(18:0/18:1/22:1)
43	TAG(12:1/22:0/22:0)	TAG(18:1/20:4/22:6)	TAG(18:1/18:1/22:0)
44	TAG(12:2/17:0/17:0)	TAG(18:2/18:2/20:2)	TAG(18:1/18:1/22:1)
45	TAG(13:0/13:0/16:0)	TAG(18:2/18:2/20:4)	TAG(18:1/20:0/20:0)
46	TAG(13:1/20:0/20:0)	TAG(18:2/18:2/20:5)	TAG(18:1/21:0/21:0)
47	TAG(14:0/14:1/22:5)	TAG(18:2/18:2/22:6)	TAG(18:1/22:1/22:1)
48	TAG(14:0/16:0/16:0)	TAG(18:2/18:3/20:5)	TAG(18:2/18:2/22:0)
49	TAG(14:0/16:0/18:1)	TAG(18:2/18:3/22:6)	TAG(20:1/20:1/22:0)
50	TAG(16:0/16:0/16:0)	TAG(18:3/18:3/22:5)	
51	TAG(16:0/16:0/17:0)		
52	TAG(16:0/16:0/18:0)		
53	TAG(16:0/17:0/18:1)		
54	TAG(16:0/18:0/18:0)		
55	TAG(16:0/18:0/18:1)		
56	TAG(16:0/18:0/22:1)		
57	TAG(16:0/18:1/22:0)		
58	TAG(16:0/20:0/20:0)		
59	TAG(16:0/22:1/22:1)		
60	TAG(16:1/16:2/20:4)		
61	TAG(16:2/16:2/16:2)		
62	TAG(17:0/17:0/19:0)		
63	TAG(17:0/17:2/19:0)		
64	TAG(17:0/18:0/18:0)		
65	TAG(17:2/17:2/18:3)		
66	TAG(18:0/18:0/18:0)		
67	TAG(18:0/18:0/20:0)		
68	TAG(18:0/18:0/20:1)		
69	TAG(18:0/18:0/22:0)		
70	TAG(18:0/18:0/22:1)		
71	TAG(18:0/18:1/20:3)		
72	TAG(18:0/18:1/21:0)		
73	TAG(18:0/18:1/22:1)		
74	TAG(18:1/18:1/20:0)		
75	TAG(18:1/18:1/22:0)		
76	TAG(18:1/18:1/22:1)		
77	TAG(18:1/20:0/20:0)		
78	TAG(18:1/21:0/21:0)		
79	TAG(18:1/22:1/22:1)		
80	TAG(18:2/18:2/22:0)		
81	TAG(19:0/19:0/19:4)		
82	TAG(20:1/20:1/20:1)		
83	TAG(20:1/20:1/22:0)		

Notes: the number of carbon chains that make up the lipid and the structure of each carbon chain is indicated in parentheses. DGTS (19:0/26:2) indicates that the diacylglyceryl trimethylhomoserine contains two carbon chains, one of which consists of 19 carbon atoms without double bonds, and the other chain consists of 26 carbon atoms containing two double bonds. PC(14:0e/20:4), e represents an ether bond in the chain structure. HexCer/NS(d18:1/16:1), d represents 2 hydroxyl groups in the chain structure. Abbreviations: Acar: acylcarnitine; AcylGlcADG: acylglucuronosyldiacylglycerol; CE: cholesteryl ester; Cer/NDS: ceramide nonhydroxy fatty acid-dihydrosphingosine; Cer/NS: ceramide nonhydroxy fatty acid-sphingosine; DAG: diacylglycerol; DGTS: diacylglyceryl trimethylhomoserine; HexCer/NS: nonhydroxy fatty acid-sphingosine; LPC: lysophosphatidylcholine; LPE: lysophosphatidylethanolamine; PC: phosphatidylcholine; SM: sphingomyelin; SHexCer: sulfur hexosylceramide hydroxy fatty acid; TAG: triacylglycerol.

## Data Availability

All data, models, and code generated or used during the study appear in the submitted article.
